# The Effect of the Integrated Chinese and Western Medicine for the Treatment of Parkinson's Disease: A Meta-Analysis

This article has been retracted.

**DOI:** 10.1155/2022/4134931

**Published:** 2022-04-08

**Authors:** Zengmian Wang, Tianshu Wang, Baoying Sheng, Weidong Song, Pengcheng Ji

**Affiliations:** ^1^Department of Neurology, The First Affiliated Hospital of Jiamusi University, Jiamusi, China; ^2^Department of Orthopaedic Surgery, The First Affiliated Hospital of Jiamusi University, Jiamusi, China; ^3^Department of Orthopaedic Surgery, The Second Affiliated Hospital of Mudanjiang Medical College, Mudanjiang, China; ^4^Department of Orthopaedic Surgery, Yakeshi Zhongmeng Hospital, Hulunbuir, China

## Abstract

**Objective:**

Traditional Chinese medicine (TCM) has been used to treat Parkinson's disease (PD), but the efficacy is still not clear. The aim of this study was to evaluate the effect of the integrated Chinese and Western medicine (ICWM) for PD through a meta-analysis.

**Methods:**

We searched randomized controlled trials comparing integrated Chinese and Western medicine (ICWM) versus conventional Western medicine (CWM) for Parkinson's disease. Data were extracted from eligible studies. We sought to evaluate pretreatment and posttreatment symptoms of PD patients and their quality of life and reduce adverse reactions. The results were expressed as risk ratio (RR) and mean difference (MD) with accompanying 95% confidence intervals.

**Results:**

Twenty-three studies were included in this study with a total of 1769 patients. The pooled results revealed that ICWM significantly improved the UPDRS score than CWM, the MD of UPDRS-I, II, III, and IV was -1.05 (95% CI: -1.42 to -0.69, *P* < 0.00001), -2.55 (95% CI: -3.19 to -1.90, *P* < 0.00001), -3.64 (95% CI: -4.69 to -2.60, *P* < 0.00001), and -0.61 (95% CI: -0.96 to -0.27, *P* = 0.0004), respectively, and ICWM also had a better score of PDQ-39 (MD = −8.71, 95% CI: -13.52 to -3.90, *P* = 0.0004) and MoCA scores (MD = 3.35, 95% CI: 1.65 to 5.04, *P* = 0.0001) compared with CWM. ICWM had certain advantages in terms of effective rate (RR = 1.27, 95% CI: 1.18 to 1.37, *P* < 0.00001) and adverse reactions (RR = 0.21, 95% CI: 0.13 to 0.36, *P* < 0.00001).

**Conclusion:**

Our research supported that ICWM had important health benefits for patients with PD and can effectively improve the symptoms of PD patients and their quality of life and reduce adverse reactions. Due to the lower quality of the included studies, large sample and multicenter randomized control test should be performed to verify our conclusions.

## 1. Introduction

Parkinson's disease (PD) is a central nervous system disease characterized by motor as the main manifestation (1). With the in-depth study of the disease, in addition to motor dysfunction, its nonmotor symptoms have also attracted attention, such as sleep disorder, anxiety and depression, cognitive dysfunction, and restless leg syndrome (2, 3). The incidence rate of common population in developed countries is about 0.3%, and the rate of people over 60 is about 1%, while it is up to 3% over 80 (4).

The treatment of PD takes compound levodopa, dopamine receptor agonist, and monoamine oxidase inhibitor as the main intervention measures (5, 6). These drugs not only alleviate the movement disorder but also play a good regulatory role in sleep. However, due to long-term use, they have side effects such as efficacy attenuation, switching phenomenon, and dyskinesia (7).

Traditional Chinese medicine (TCM) believes that PD belongs to “vibration disease,” and those with muscle tension, spasm, and slowness of movement can be diagnosed as TCM detention disease; those with both obvious symptoms can be diagnosed as “shaking detention disease” in TCM (8). TCM uses the combination of disease and syndrome, syndrome differentiation, treatment according to syndrome, and other methods to treat PD and has achieved good clinical effects in terms of increasing efficiency and reducing toxicity and improving the patients' quality of life (9). TCM is a holistic medical system, which includes herbal medicine, acupuncture, tai chi, massage, diet therapy, and qigong. Many studies have found that the combination of traditional Chinese medicine and Western medicine has both synergistic efficacy and the advantages of reducing the adverse reactions of Western medicine (10, 11).

So far, a large number of studies have been carried out to study the role of the integrated Chinese and Western medicine (ICWM) in the treatment of PD (12, 13). In view of the lack of relevant systematic evaluation, this study was aimed at comprehensively collecting the published randomized controlled trials (RCTs) of the ICWM for the treatment of PD and systematically evaluating the stability and safety of its efficacy by comparing the clinical efficacy of the ICWM and conventional Western medicine (CWM) in the treatment of PD, so as to provide basis for rational and safe drug use.

## 2. Methods

### 2.1. Literature Search Strategy

Two authors (Z Wang and T Wang) performed a systematic search in 6 electronic databases including Cochrane Central Register (CENTRAL), PubMed, China National Knowledge Internet (CNKI) Database, Chinese Biological Medical (CBM) Database, Wanfang Database, and China Science and Technology Journal Database (VIP) (up to December 31, 2021) with the following keywords: (1) traditional Chinese medicine; (2) Chinese medicine; (3) Parkinson's disease; and (4) Parkinsonism. The search strategy was refined by combining the keywords using the Boolean operators “OR” or “AND.” There were no restrictions on the publication language in the literature search. Disagreements were resolved through consensus between the reviewers.

### 2.2. Study Selection

Inclusion criteria included the following: (1) researches comparing patients who receive integrated Chinese and Western medicine (ICWM) with conventional Western medicine (CWM); (2) patients with Parkinson's disease; (3) containing indicators evaluating effectiveness between the two therapy; and (4) available in full text. The exclusion criteria were as follows: (1) ineligible article design; (2) duplicate articles; (3) reviews, protocols, or letters; and (4) no sufficient related outcomes.

### 2.3. Data Extraction and Quality Assessment

Two independent reviewers (B Sheng and W Song) performed the study selection, quality assessment, and data extraction. All available information related to our study topic was extracted from the included studies, including study authors, study design, treatment therapy, patients' characteristics (age and gender), year of outset, and time of follow-up.

We assessed the methodological quality of the included studies by the Cochrane Collaboration tool, which was based on the following six items: allocation concealment, random sequence generation, blinding (objective outcomes), blinding (self-reported), selective and incomplete outcome reporting, and other bias presence.

### 2.4. Statistical Analysis

All statistical analyses were performed by using Review Manager (version 5.4) software (RevMan; The Nordic Cochrane Centre, Copenhagen, Denmark, 2020). Continuous variables were expressed as mean difference (MD) with 95% confidence interval (CI), and risk ratio (RR) was used for classification data. Heterogeneity of the data was assessed using the chi test and *I*^2^ values. *I*^2^ of 25, 50 and 75% will be considered to represent low, medium, and high heterogeneity, respectively. A fixed effect model was applied in the absence of heterogeneity, while random effect model was used if heterogeneity was observed. Publication bias was evaluated by visual inspection of funnel plots and using Egger's tests.

## 3. Results

### 3.1. Search Process

A total of 326 eligible studies were screened. After exclusion of 303 trials that did not meet our inclusion criteria, 23 randomized RCTs with a total of 1769 patients were included (14–36). The process of literature retrieval is shown in Figure 1.

### 3.2. Characteristics of the Included Studies

Table 1 showed the main characteristics of the included studies. The ICWM group treatment contained herbal prescription, decoction, capsule, and granule, and the CWM group was treated with medoba, donepezil, levodopa, or dopashydrazine. All these studies were published from 2011 to 2021. The sample size ranged from 24 to 120.

### 3.3. Results of the Quality Assessment

The quality of the included studies were assessed in accordance with Cochrane Collaboration tool. There were no high risk of six kinds of bias in each studies (Figure 2). A summary of the risk of bias assessment for all included studies is shown in Figure 3.

### 3.4. Results of the Heterogeneity Test

#### 3.4.1. UPDRS Score

The Parkinson's disease rating scale (UPDRS) scored the patient's condition before and after treatment and evaluated the scores of four parts of UPDRS: I, II, III, and IV. Part I mainly evaluated the patient's mental behavior and emotional factors, part II evaluated the patient's ability of daily living, part III evaluated the patient's motor ability, and part IV evaluated the complications during treatment. Ten, eleven, twelve, and eight trials compared the effect of the ICWM versus CWM according to changes in the UPDRS-I, II, III, and IV score, respectively.

The pooled results from the random effect model showed that the ICWM group had a higher decrease of UPDRS-I, II, III, and IV than the CWM group, as the MD of UPDRS-I, II, III, and IV were -1.05 (95% CI: -1.42 to -0.69, *P* < 0.00001), -2.55 (95% CI: -3.19 to -1.90, *P* < 0.00001), -3.64 (95% CI: -4.69 to -2.60, *P* < 0.00001), and -0.61 (95% CI: -0.96 to -0.27, *P* = 0.0004), respectively (Figure 4). The results demonstrated that ICWM showed a significant beneficial effect in improving mental behavior, emotional factors, ability of daily living, motor ability, and complications than CWM.

#### 3.4.2. PDQ-39 Score

Six studies involving 430 patients contributed to the analysis of life quality, by using the questionnaires of the 39-item Parkinson's disease questionnaire (PDQ-39). The pooled analysis indicated that, compared with CWM group, the ICWM group resulted in a great improvement in the PDQ-39 score with a MD of -8.71 (95% CI: -13.52 to -3.90, *P* = 0.0004; Figure 5). However, significant heterogeneity among the studies was detected (*I*^2^ = 99%, *P* < 0.00001).

#### 3.4.3. Cognitive Function

For cognitive function, three studies contained 236 patients reported it by the instruments of the Montreal Cognitive Assessment (MoCA). The MoCA scores of the ICWM group was significantly higher than the CWM group (MD = 3.35, 95% CI: 1.65 to 5.04, *P* = 0.0001; Figure 6).

#### 3.4.4. Effective Rate

In the evaluation of difference of effective rate between the ICWM group and CWM group, ten articles which involved 770 patients were selected. The pooled analysis showed that compared to the CWM group, the ICWM group had a better level of effective rate (RR = 1.27, 95% CI: 1.18 to 1.37, *P* < 0.00001) (Figure 7), without significant heterogeneity (*I*^2^ = 36%, *P* = 0.12) (Figure 7).

#### 3.4.5. Adverse Reaction

A total of eight studies reported the adverse reaction. The forest plot showed that the rate of adverse reactions in the ICWM group was lower than CWM group (RR = 0.21, 95% CI: 0.13 to 0.36, *P* < 0.00001) (Figure 8), without significant heterogeneity among studies (*I*^2^ = 0%, *P* = 0.81) (Figure 8).

### 3.5. Publication Bias

Funnel plots were performed to evaluate the publication bias. Two funnel plots were produced for indexes of effective rate and adverse reaction, and they showed some evidence of asymmetry (Figure 9), but the Egger's linear regression for quantitative publication bias of two indexes was nonsignificant (effective rate, *P* = 0.478; adverse reaction, *P* = 0.751), which suggested that no significant publication bias existed in our meta-analysis.

## 4. Discussion

With the increasing global aging society, the prevalence and incidence of PD continue to increase. Studies have confirmed that almost all PD patients have at least one nonmotor symptom, which is closely related to the duration of PD, disease severity, and cognitive function (37). Damage is closely related, which is also the main factor affecting the quality of life of patients and even late disability. In terms of Western medicine treatment, levodopa is still the only reported drug that can prolong life expectancy, but after long-term replacement therapy treatment, it will become less and less advantageous, and more than 50% of PD patients will eventually experience severe movement disorders, sleep attacks, and adverse reactions, resulting in an immeasurable burden on patients, families, and society (38, 39). Traditional Chinese medicine is effective in alleviating various symptoms, especially age-related symptoms.

Compared with the traditional CWM, ICWM treatment can prolong the increase of CWM dosage and the time course of combined medication. At the same time, traditional Chinese medicine has less toxic and side effects (40). Therefore, taking advantage of the traditional Chinese medicine can not only improve the clinical symptom severity score of PD but also have fewer adverse reactions (41, 42).

The results of this study showed that the treatment of PD with ICWM was better than the simple CWM treatment in reducing the UPDRS score and improving the PDQ-39 (MD = −8.71, 95% CI: -13.52 to -3.90, *P* = 0.0004), and it was also better than CWM in the MoCA scores (MD = 3.35, 95% CI: 1.65 to 5.04, *P* = 0.0001). There are certain advantages in terms of effective rate (RR = 1.27, 95% CI: 1.18 to 1.37, *P* < 0.00001) and adverse reactions (RR = 0.21, 95% CI: 0.13 to 0.36, *P* < 0.00001). This is consistent with Tian's research results (43).

This meta-analysis has the following limitations. First, most of the included studies were in Chinese, with only 3 articles in English, and the research subjects were all domestic patients. There may be bias in population selection and low research quality. Second, only 6 of the included studies used a random number table, and the rest of the studies mentioned “random” but did not specify the random method. Third, except for 3 studies that adopted double-blind method, the rest did not mention the specific blinding method. Fourth, sleep disorders in PD require long-term treatment, and the included studies lack long-term follow-up.

To sum up, ICWM can effectively improve the symptoms of PD patients and their quality of life and reduce adverse reactions. It is a safe and effective intervention method in clinical practice. Due to the limitations of the quality and quantity of the included studies, this systematic review still has many deficiencies. More randomized controlled trials should be implemented to further strengthen this evidence.

## Figures and Tables

**Figure 1:** Flowchart of the literature search and study selection.

**Figure 2:** Quality assessment of the included studies: low risk (green), unclear (yellow), and high risk (red).

**Figure 3:** Quality assessment of the included studies: low risk (green), unclear (yellow), and high risk (red).

**Figure 4:** Forest plot showing the mean difference in the UPDRS score between ICWM and CWM groups.

**Figure 5:** Forest plot showing the mean difference in the PDQ-39 score between ICWM and CWM groups.

**Figure 6:** Forest plot showing the mean difference in the cognitive function between ICWM and CWM groups.

**Figure 7:** Forest plot showing the risk ratio in the effective rate between ICWM and CWM groups.

**Figure 8:** Forest plot showing the risk ratio in the adverse reaction between ICWM and CWM groups.

**Figure 9:** Funnel plot for publication bias in this meta-analysis. (a) Effective rate and (b) adverse reaction.

**Table 1:** Clinical baseline information and primary conclusion of studies.

Study	Study design	Treatment		No. of patients		Gender (M/F)		Age		Follow-up	Duration
		Intervention	Control	Intervention	Control	Intervention	Control	Intervention	Control		
Li Chengdong 2011	RCT	Herbal fumigation and washing prescription+medoba	Medoba	40	40	23/17	24/16	61 ± 11.83	61 ± 11.83	4 months	2006 to 2010
Wan Fung Kum 2011	RCT	Jia Wei Liu Jun Zi Tang+CMW	CMW	22	25	14/8	17/8	64.82 ± 8.88	60.88 ± 9.41	24 weeks	NR
Weidong Pan 2011	RCT	Zeng-xiao An-shen Zhi-chan 2+CMW	CMW	56	54	34/22	32/22	62.82 ± 10.31	63.1 ± 10.2	13 weeks	2008 to 2010
Yang Qingtang 2012	RCT	Shaoyao Gancao decoction+Ganmai Dazao decoction+medoba	Medoba	34	34	NR	NR	45-80	45-80	12 weeks	2009 to 2011
Yu Dengjun 2012	RCT	Ginseng Guipi decoction+medoba	Medoba	50	48	NR	NR	70.02 ± 6.73	70.02 ± 6.73	4 weeks	2009 to 2011
Zhong Cheng 2012	RCT	Bushen Huoxue Tongluo capsule+CMW	CMW	60	60	NR	NR	51-82	51-82	3 months	2011 to 2012
Chen Mengyun 2014	RCT	Zhizhan granule+CMW	CMW	57	51	38/19	35/16	66.44 ± 7.64	65.63 ± 7.37	12 weeks	2012 to 2013
Chao Gu 2015	RCT	Di-Huang-Yi-Zhi+donepezil	Donepezil	30	30	14/16	13/17	67.33 ± 9.31	67.06 ± 9.63	6 months	2010 to 2013
Wen Lili 2015	RCT	Cistanche wuxifeng granule+medoba	Medoba	29	28	15/14	16/12	70.79 ± 7.50	71.21 ± 5.95	3 months	2013 to 2014
You Jiahua 2015	RCT	Shujin dingzhan decoction+CMW	CMW	30	30	22/8	20/10	65.4 ± 7.9	65.1 ± 8.2	12 weeks	2013 to 2014
Bai Yu 2016	RCT	Zishen RouJing decoction + CMW	CMW	54	54	33/21	35/19	66.81 ± 7.86	66.16 ± 7.72	12 weeks	2007 to 2015
Xu Qingshui 2016	RCT	Cistanche Rongjing+levodopa	Levodopa	14	10	8/6	7/3	60.35 ± 8.17	63.22 ± 6.79	3 months	NR
Ye Qing 2016	RCT	Yizhi Pingzhan recipe+levodopa	Levodopa	40	38	25/15	23/15	67.59 ± 7.89	65.93 ± 6.63	3 months	2013 to 2015
Zhang Lijuan 2016	RCT	Qingxin Kaiqiao recipe+acupuncture+medoba	Medoba	49	49	NR	NR	62.3 ± 11.2	63.1 ± 10.5	4 months	2015
Cai Li 2017	RCT	Zhizhan decoction+CMW	CMW	43	43	25/18	23/20	57.24 ± 3.36	58.14 ± 4.12	12 weeks	2014 to 2016
Chen Yu 2017	RCT	Tianma goutengyin and Shaoyao Gancao decoction+medoba	Medoba	36	36	22/14	21/15	68.8 ± 10.5	67.7 ± 9.9	3 months	2013 to 2015
Wang Jiecheng 2017	RCT	Self-made prescription+dopashydrazine	Dopashydrazine	49	49	28/21	25/24	72.32 ± 10.72	73.81 ± 10.64	4 weeks	2016
Mo Haizhen 2018	RCT	Yishen tiaogan Jieyu recipe+dopashydrazine	Dopashydrazine	30	30	13/17	11/19	62.74 ± 4.89	64.57 ± 6.68	8 weeks	2016 to 2017
Xu Xiao 2018	RCT	Shaoyao Gancao decoction+CMW	CMW	30	30	16/14	17/13	52 ± 11.32	53 ± 11.45	3 months	2014 to 2017
Cao Jianfeng 2020	RCT	Dialectical prescription+levodopa	Levodopa	45	45	29/16	28/17	68.56 ± 2.71	68.63 ± 2.62	8 weeks	2016 to 2018
Liao Xun 2020	RCT	Dialectical prescription+dopashydrazine	Dopashydrazine	36	36	20/16	18/18	52.47 ± 1.36	51.42 ± 1.48	11 weeks	2018 to 2019
Zhao Lili 2020	RCT	Dialectical prescription+medoba	Medoba	60	15	NR	NR	NR	NR	5 weeks	2017 to 2019
Zhang Quan 2021	RCT	Yangxue Pinggan granule+CMW	CMW	20	20	10/10	11/9	57.00 ± 13.87	58.00 ± 14.05	8 weeks	2017 to 2019

RCT: randomized controlled trail; CMW: conventional Western medicine; NR: not reported.

## Data Availability

No data were used to support this study.
